# Mechanisms and Drug Intervention for Doxorubicin-Induced Cardiotoxicity Based on Mitochondrial Bioenergetics

**DOI:** 10.1155/2022/7176282

**Published:** 2022-10-14

**Authors:** Guanjing Ling, Xiaoping Wang, Nannan Tan, Jing Cao, Weili Li, Yawen Zhang, Jinchi Jiang, Qianbin Sun, Yanyan Jiang, Wei Wang, Yong Wang

**Affiliations:** ^1^School of Chinese Medicine, Beijing University of Chinese Medicine, Beijing 100029, China; ^2^School of Life Sciences, Beijing University of Chinese Medicine, Beijing 100029, China; ^3^Beijing Key Laboratory of TCM Syndrome and Formula, Beijing 100029, China; ^4^Key Laboratory of Beijing University of Chinese Medicine, Ministry of Education, Beijing 100029, China; ^5^Guangzhou University of Chinese Medicine, Guangzhou 510006, China

## Abstract

Doxorubicin (DOX) is an anthracycline chemotherapy drug, which is indispensable in antitumor therapy. However, its subsequent induction of cardiovascular disease (CVD) has become the primary cause of mortality in cancer survivors. Accumulating evidence has demonstrated that cardiac mitochondrial bioenergetics changes have become a significant marker for doxorubicin-induced cardiotoxicity (DIC). Here, we mainly summarize the related mechanisms of DOX-induced cardiac mitochondrial bioenergetics disorders reported in recent years, including mitochondrial substrate metabolism, the mitochondrial respiratory chain, myocardial ATP storage and utilization, and other mechanisms affecting mitochondrial bioenergetics. In addition, intervention for DOX-induced cardiac mitochondrial bioenergetics disorders using chemical drugs and traditional herbal medicine is also summarized, which will provide a comprehensive process to study and develop more appropriate therapeutic strategies for DIC.

## 1. Introduction

With continuing development of medical technology and increasing improvements in tumorous diagnoses, the lifespans of patients with malignant tumours have been significantly prolonged. However, morbidity and mortality from complications caused by anticancer therapy are increasing year by year, among which cardiovascular disease (CVD) has become the main cause of death for cancer survivors. It has been reported that approximately 20%~30% of cancer patients die due to CVD [1, 2]. In this situation, cardio-oncology as a new field has come into being. Doxorubicin (DOX), an anthracycline chemotherapeutic drug, is indispensable in antitumor therapy. Low doses of DOX are effective in treating various cancers. However, accumulating doses of doxorubicin can induce severe cardiotoxicity (DIC), which largely limits its application [3]. DIC is clinically characterized by increased ventricular wall thickness, decreased left ventricular ejection fraction, arrhythmias, and heart failure, finally leading to death [4, 5]. To date, the most widely accepted hypothesis for DIC is that the DOX quinone moiety, oxygen molecules, and other cellular electron donors make an electronic exchange to generate excessive reactive oxygen species (ROS). DOX can also undergo redox cycling, and then generate oxygen radicals by forming complexes with iron. Although increased ROS production in cardiomyocytes after DOX therapy has been confirmed in vivo and in vitro, antioxidants and iron chelation both cannot prevent DIC. Collectively, although massive effort is to be made in identifying strategies to prevent DIC, a satisfying approach is lacking [6–9].

Heart is a high-energy-consuming organ that requires a large amount of ATP every day to ensure its normal physiological function [10]. In healthy adult hearts almost all ATP is produced by the oxidative metabolism of mitochondria. Drugs that interfere with mitochondrial function may lead to the exhaustion of ATP, and finally leading to myocardial dysfunction. Mitochondrial bioenergetics is related to myocardial substrate utilization, the mitochondrial respiratory chain, high-energy phosphate storage, transport and energy signalling pathways, and other processes related to mitochondrial structure and function. It has been reported that DOX-induced mitochondrial bioenergetic collapse (DiMBc) may be mediated in numerous ways: by damaging the Krebs cycle, fatty acid *β*-oxidation, the respiratory chain, and oxidative phosphorylation, resulting in a bioenergy crisis that ultimately leads to cardiomyocyte necrosis [11–13]. Mechanistically, mitochondrial bioenergetic collapse has become a significant feature of DIC, whether at an early stage, intermediate stages, or in the long-term [14]. Understanding the mechanisms of DiMBc could help identify new targets to develop novel strategies for preventing DIC in cancer patients. Herein, we concentrated on describing the molecular processes regulating mitochondrial bioenergy whose dysregulation has been linked to DIC. DOX interferes with cardiac bioenergy production at multiple levels by affecting cardiac mitochondrial substrate metabolism, ATP storage and utilization, mitochondrial respiratory chain function, and a range of metabolically related targets (Figure 1). In an hPC-CM model system, a GO analysis centred on genes that involved in DNA damage, ROS generation, and mitochondrial pathway showed powerful evidence of upregulation of these pathways by DOX [15]. Although some molecular mechanisms have not yet been absolutely established, mitochondrial bioenergy metabolism plays an important role in DIC according to current studies. Further study of this mechanism and the development of drugs targeting these targets are expected to provide more and better options for improving DIC. Moreover, we discuss how the determination of key players in mitochondrial bioenergy is instrumental to refining current relevant achievements in drug intervention for DiMBc.

## 2. Myocardial Mitochondrial Substrate Metabolism

In normal myocardium, approximately 60%~90% of energy comes from mitochondrial fatty acid *β*-oxidation, with a limited amount coming from glucose metabolism [16]. The oxidation of fatty acids is similar to glucose oxidation: both undergo a series of oxidative decarboxylation reactions to produce acetyl-CoA and NADH/FADH_2_, after which the former enters the Krebs cycle (TCA cycle), and the latter participates in electron transfer in the mitochondrial respiratory chain to produce a large quantity of ATP [17]. DOX mediates cardiotoxicity by affecting myocardial bioenergy generation at multiple levels of myocardial substrate metabolism. Mechanistically, DOX has been proved to impact gene expression involved in anaerobic glycolysis and aerobic fatty acid oxidation (FAO). Recently, DOX-related DNA transcription obstruction has also been related to mitochondrial dysfunction. It is speculated that the early metabolic changes of the heart in DIC may be related to systemic DNA damage [18, 19]. (Figure 2).

Evidence demonstrates that heart energy mainly comes from fatty acid *β*-oxidation metabolism in the presence of oxygen. Moreover, it has been reported that DOX treatment causes a significant increase in plasma and cardiac total cholesterol, triglycerides, high-density lipoproteins, and low-density lipoproteins in animal models [20–22]. Therefore, systemic lipid indicators are considered attractive predictors for long-term cardiovascular events, which need to be further validated. Thereafter, statins, as lipid-lowering drugs, can inhibit the activity of *β*-hydroxy-*β*-methylglutaryl CoA (HMG-CoA) reductase, thereby reducing the production and utilization of cholesterol and ultimately leading to the reduction of blood lipids, thus reducing coronary atherosclerosis and other cardiovascular events in patients [23, 24]. In addition, statins can act on Rac1, an indispensable subunit of NADPH oxidase and necessary for its activity. DOX induces DIC through Rac1 in both ROS-dependent and ROS-independent p53 pathways. Statins inhibit Rac1 activation, thereby alleviating DIC [25]. In addition, peroxisome proliferator-activated receptors (PPARs), which are ligand-activated transcription factors, can control the expression of genes involved in lipid metabolism and inflammation [12]. Studies have shown that DOX significantly downregulates the mRNA or protein levels of PPARs, thereby affecting the expression of corresponding target genes [26–28]. PPAR*γ* agonists significantly reduce serum TAG, suggesting that DOX may inhibit the expression or activity of target genes such as lipoprotein lipase (LPL) by inhibiting PPAR*γ* to inhibit the hydrolysis of TAG and uptake into tissue cells [28–30]. However, some studies have indicated that DOX significantly reduces the content of myocardial triglyceride (TAG) but does not affect the expression or phosphorylation of enzymes related to TAG catabolism and storage such as hormone-sensitive lipase (HSL), adipose triglyceride lipase (ATGL), and perilipin 5 (PLIN5). Importantly, ATGL overexpression further reduces TAG levels but improves cardiac function. It is suggested that DOX reduces the myocardial TAG level by reducing the uptake of cardiac fatty acids and the synthesis of new TAGs rather than increasing the catabolism of TAGs, and this is an adaptive response which may also be related to DOX inhibition of PPARs [31].

Fatty acids need to enter cells before they can be oxidized. Human leukocyte differentiation antigen 36 (CD36), also described as fatty acid translocase (FAT), is a transmembrane transport glycoprotein and an important transporter of fatty acid uptake in cardiac tissue. It is closely related to fatty acid metabolism [32]. It has been documented that DOX can downregulate CD36 mRNA levels thereby reducing myocardial fatty acid uptake and oxidative metabolism as well as fatty acid resynthesis of TAG in myocardial tissue. This may be related to the downregulation of PPAR levels by DOX, since CD36 is a known target gene of PPARs [33]. After entering the cell, fatty acids are activated in the cytoplasm to form acyl-CoA, and then enter the mitochondria for *β* oxidation. Activated fatty acids need to be transported to mitochondria by carnitine palmitoyl transferase 1/2 (CPT 1/2) in the presence of L-carnitine, a rate-limiting step in FAO, and these enzymes are key to FAO. Studies have reported that DOX treatment significantly reduces the activity of CPT1/2 and inhibits the oxidation of fatty acids while supplementation with L-carnitine restores the oxidation level of fatty acids but does not improve the activity of CPT1/2. It is suggested that DOX may disrupt fatty acid entry into mitochondria by disrupting CPT1/2 activity or depleting L-carnitine leading to a decrease in FAO [34–37].

A small part of the energy required by the heart comes from glucose metabolism. Similarly, glucose needs to enter the cell, mediated by glucose transporter 1 (GLUT1) on the cell membrane [10]. It has been shown that early DOX treatment significantly increases and subsequently decreases myocardial glucose uptake. Consistent with this, DOX treatment quickly promotes the recruitment of myocardial GLUT1 to the membrane without affecting its overall level, suggesting that the early increase in glucose uptake induced by DOX treatment is an adaptive response to myocardial energy deficiency [38]. In addition, DOX treatment can lead to long-term restriction of glycolysis, which may be related to DOX lowering the mRNA levels of hexokinase 2 (HK2) and phosphofructokinase (PFK), which are known key enzymes in glycolysis [39].

AMP-activated protein kinase (AMPK), a cellular energy sensing centre, can be activated in response to energy deprivation and modulates its downstream targets to increase ATP production [40, 41]. Activation of AMPK has beneficial effects on mitochondria, triggering catabolic pathways such as FAO metabolism and glycolysis, and downregulating anabolism, which is mainly mediated by the mTOR signalling pathway [39]. AMPK can increase oxidative mitochondrial metabolism via activation of PGC-1*α* signalling, decrease apoptosis via inhibition of mTOR signalling, and directly or indirectly increase autophagy via activation of mammalian Unc-51 like autophagy activating kinase (ULK1) or inhibition of mTOR signalling [42, 43]. AMPK is therefore the key target for many mechanisms involved in DIC, and cardiac AMPK signalling pathway has been demonstrated to be impaired by DOX. Experimental evidence shows that a DOX-mediated decrease in p-AMPK levels drives metabolic disarrangements and cellular substrate overload. Furthermore, DOX may activate mTOR through the inhibition of AMPK and the activation of Akt/ERK, resulting in a reduction in glycolipid oxidation levels and an increase in ATP consumption. Studies suggest that inhibition of AMPK by DOX may be mediated by crosstalk with the Akt/ERK signalling pathway, and Akt inhibitors can reverse DOX inhibition of AMPK [44]. Acetyl-CoA carboxylase (ACC), an enzyme which is directly inhibited by AMPK, is overactivated to catalyse the formation of malonyl-CoA, irreversibly inhibiting CPT1 and FAO [45, 46]. In addition, according to the report, the DOX can promote the migration of CD11b^+^ macrophages from the peripheral blood to the heart and release interferon *γ* (IFN*γ*), interfering with normal mitochondrial respiration and FAO of cardiomyocytes by inhibiting the AMPK/ACC axis depending on the p38 branch, linking inflammatory signalling, metabolic remodelling, and DIC [47, 48]. The renin-angiotensin system is the core factor regulating blood pressure and electrolytes. Clinical studies have discovered that angiotensin II (Ang II) type 1 receptor (AT1R) antagonists can prevent cardiovascular events. Studies have confirmed that Ang II can activate AMPK by stimulating NADPH oxidase and inducing reactive oxygen species production. DOX significantly increases Ang II levels, suggesting that DOX may activate AMPK through upregulation of Ang II levels [49–51]. Leptin is a cytokine-like hormone that can be produced in the heart. An increasing number of studies have shown that leptin regulates energy homeostasis through a direct effect of peripheral lipids and glucose metabolism. Studies have shown that in mice with diet-induced obesity (DIO), an increase in leptin can promote an increase in AMPK phosphorylation, which leads to an increase in FAO. It is known that DOX treatment increases cardiac leptin levels, suggesting that DOX may also promote AMPK phosphorylation through the upregulation of leptin. The exact mechanisms need to be further confirmed [52–54]. The restoration of AMPK activity makes a beneficial impact on mitochondria, reducing oxidative stress and maintaining mitochondrial energy production against DIC [42]. Collectively, this evidence indicates that AMPK plays a pivotal role in DiMBc and regulates cardiac metabolic remodelling by interacting with energy metabolism-related targets. The development of drugs targeting these metabolism-related proteins of cardiac substrates is a promising direction.

DOX has also been reported to reduce citrate synthase (CS) activity, thereby affecting the TCA cycle [55]. DOX also interferes with the expression of many cardiac genes, in particular downregulating genes for several enzymes involved in energy metabolism, including enzymes in relation to mitochondrial oxidative phosphorylation such as iron-sulfur Protein, cytochrome c oxidase, phosphofructokinase, energy transfer enzyme (MCK), and adenylate kinase AK3 [56]. In addition, in clinical studies, patients with DIC have shown changes in citric acid and aconitine, and the plasma levels of purine and pyrimidine metabolites underwent significant changes [57]. These results indicate that DOX can affect multiple levels and targets in myocardial substrate metabolism, suggesting that substrate metabolism is an important mechanism and treatment direction for DIC.

## 3. Myocardial Mitochondrial Respiratory Chain and Storage/Utilization of ATP

The reductive equivalents generated by substrate metabolism are transferred sequentially between four main multienzyme complexes in the inner membrane of mitochondria, in which CI and CII are coupled with a proton pump, and electron transfer is accompanied by hydrogen proton transfer from the mitochondrial matrix to the intermembrane space [58]. Finally, cytochrome aa3 (Cytaa3) transfers electrons from cytochrome c (Cytc) to oxygen molecules to form reactive oxygen species, which can combine with hydrogen protons to generate H_2_O. The electrochemical gradient generated on the mitochondrial membrane provides the essential free energy for ATP synthase to catalyse the synthesis of ATP from ADP and Pi [59]. ATP transfer is achieved through the energy shuttle mechanism of creatine kinase, an enzyme that delivers energy to cardiac myofibrils for utilization [60]. (Figure 3).

Cardiolipin is an important component of the inner mitochondrial membrane and is necessary for the activities of the enzymes of respiratory chain such as cytochrome c oxidase [61]. Cytc, a small water-soluble protein, is involved in the formation of respiratory chain complexes as an electron transporter. Cardiolipin binds to it under electrostatic action thereby promoting the conformational change of its prosthetic group haem catalytic centre to form Cytc oxidoreductase. DOX has a strong affinity for cardiolipin, and its specific irreversible binding prevents cardiolipin from acting as a cofactor of the respiratory chain complex, destroying the activity of CI, CIII, and CIV that require cytochromes in the electron transport chain (ETC), leading to ROS excessive generation and ATP synthesis disorder [62]. This also leads to the loss of normal function in cardiolipin-dependent inorganic phosphate carriers and mtCK, inhibiting oxidative phosphorylation and the storage and utilization of ATP [63]. In addition, cardiolipin is structurally or functionally related to ANT and VDAC involved in the formation of the mitochondrial permeability conversion pore (mPTP). Studies have shown that DOX binding to cardiolipin can also promote the opening of mPTP, resulting in content leakage and loss of mitochondrial structure and function [39].

Mitochondrial respiratory chain CI can catalyse the reduction of DOX to the semiquinone type, which forms ROS or RNS in redox cycling, further damaging the mitochondrial respiratory chain [64, 65]. RNS mainly causes myocardial damage through the rapid reaction of NO and superoxide to nitrite, such as inhibiting creatine kinase, interfering with cell calcium circulation, and affecting mitochondrial function [66, 67]. DOX binds to DNA topoisomerase II*β* (TOPII*β*) and DNA in cardiomyocytes to form a term-cracking complex, downregulating the expression of Ndufa3, Sdha, and Atp5a1 involved in the ETC; inducing mitochondrial ultrastructure and function changes; and exacerbating mitochondrial dysfunction and ROS formation [56, 68, 69]. DOX interferes with complex IV subunit 1 and uncoupling protein 3 (COXI-UCP3) coupling through Bcl-2/19-kDa interaction protein 3 (Bnip3), resulting in mitochondrial membrane potential loss and inhibition of normal mitochondrial respiration [70]. In vivo and in vitro animal experiments have proved that DOX destroys the activity of mitochondrial respiratory chain-related enzymes through a variety of mechanisms, disrupting the generation of myocardial energy. Additionally, the destruction of the mitochondrial respiratory chain is closely related to the generation of ROS, and the two interact with each other to further aggravate myocardial injury.

Phosphocreatine is the stored form of energy in the heart. Under the action of creatine kinase, creatine is converted to phosphocreatine, powered by ATP. When ATP is insufficient, phosphocreatine can break down and release energy to promote the phosphorylation of ADP to ATP. Studies have shown that DOX may downregulate the CK level, reducing the phosphocreatine to creatine ratio, which results in changes in mitochondrial creatine kinase activity [71]. Only the CK-MB isozyme of creatine kinase is expressed in cardiac tissue, and DOX can react with Fe^2+^, resulting in the oxidative damage of creatine isozyme, thus destroying the utilization of ATP by cardiac cells [72, 73]. These results suggest that drugs targeting the CK system may play a significant role in preserving the heart from DIC.

## 4. Other Mechanisms by which DOX Affects Myocardial Mitochondrial Bioenergy

DOX can not only affect processes such as myocardial substrate utilization, mitochondrial respiratory chain, high-energy phosphate storage, and transport but also directly destroy mitochondrial structure and quantity through other mechanisms, resulting in mitochondrial bioenergetic collapse. (Figure 4).

### 4.1. Mitochondrial Permeability Transition Pore (mPTP) Opening

Mitochondrial permeability conversion (mPT) is a pathophysiological state of the mitochondrial intima (IMM), mainly realized through the mPT pore (mPTP). mPTP is a protein complex which is located between the outer and inner membranes of mitochondria. ANT, VDAC, and CypD are believed to be involved in the formation or regulation of mPTP. ANT is an adenine nucleotide (ADP/ATP) translocator involved in the exchange of cytoplasmic ADP and mitochondrial ATP [73]. Although it is controversial whether ANT is an essential component of mPTP, it undeniably plays a crucial role in regulating the activity of mPTP [74, 75]. DOX reduces the ANT content of cardiac mitochondria, resulting in increased mPTP opening, mitochondrial fragmentation, and reduced respiration [76, 77]. Cyclophilin D (CypD) is also a functional regulator of mPTP, and impaired NF-*κ*B signalling is the basis of CypD-mediated mPTP opening in DIC. Nuclear factor-kappa B (NF-*κ*B) is a transcriptional repressor of the mitochondrial death protein Bnip3. DOX can inhibit NF-*κ*B, thereby activating Bnip3 and localizing to mitochondria through its carboxy-terminal transmembrane domain (TM). mPTP opening is mediated by the formation of protein complexes with CypD, resulting in the loss of mitochondrial membrane potential and the raising in ROS production. It may be proved beneficial to maintain NF-*κ*B signalling in reducing mitochondrial dysfunction in DIC, while the protection offered by NF-*κ*B may be temporary [70, 78]. Another major trigger for mPTP opening is mitochondrial calcium (Ca^2+^) overload. Mitochondrial matrix Ca^2+^ regulates basic cellular processes such as energy metabolism. The biological basis of mitochondrial Ca^2+^ homeostasis has received extensive attention owing to the calcium dysregulation characteristic of impaired mitochondrial bioenergetics and cardiomyocyte death in DIC [79]. It has been given evidence that DOX triggers the RIP3-mediated activation of CaMKII, leading to mPTP opening and myocardial necroptosis [80]. In addition, DOX stimulates mPTP opening by weakening the binding of phospho-GSK-3*β* (Ser9) to ANT [81]. In addition, DOX also activates acidic sphingomyelinase, which contributes to ceramide accumulation, thereby coupling volt-independent B-type calcium channel activity with mPTP opening [82]. The mPTP is also thought to be a common pathway leading to many types of cell death such as apoptosis, necrosis, and ferroptosis. Importantly, mPTP is identified as the primary target of DOX-induced iron-dependent death acting on isolated mitochondria. mPTP protectors can counteract iron-DOX complex-induced Ca^2+^-dependent mPTP opening [74]. These data offer new treatment options to the modulation of the toxic influence of DOX on mitochondria by reducing their dysfunction. In addition, DOX upregulates the expression of the proapoptotic proteins BAX and BAK, mediating the opening of mPTP and the release of Cytc and AIF and causing significant mitochondrial morphological disorders, including crest loss and mitochondrial fragmentation, which ultimately leads to mitochondrial bioenergy disorders [5]. Mitochondrial phosphate carrier (PiC) is the main pathway of mitochondrial phosphate transmembrane transport and acts as a regulator of mPTP, promoting mPTP opening and Cytc release. A recent finding shows that prolonged doxorubicin treatment significantly increases phosphate carrier protein expression [83]. In summary, DIC is thought to be mediated partly via disruption of mitochondrial function, increased opening of the mPTP, and the release of Cytc, resulting in myocyte apoptosis and disruption of mitochondrial bioenergetics.

### 4.2. Mitochondrial DNA (mtDNA) Damage

Each cardiomyocyte has thousands of mitochondria with their own DNA, called mitochondrial DNA (mtDNA), which can encode multiple proteins in the mitochondrial respiratory chain [84]. Topoisomerase II (TOPII) can cleave two strands of DNA and untie the superhelix structure of DNA double strands, playing an important role in gene replication and transcription. There are two TOPII types: TOPII*α* and TOPII*β*. TOPII*α*, a known marker for cell proliferation, is overexpressed in tumour cells, while only TOPII*β* expression has been detected in cardiomyocyte mitochondria [85, 86]. One target of DOX is TOPII. In tumour cells, DOX binds DNA and TOPII to form a ternary division complex that causes tumour cell death, the molecular basis of DOX anticancer activity. DOX can also form a terpolymer complex with TOPII*β*-DNA in normal hearts to induce DNA double-strand breaks (DSBs) leading to cardiomyocyte death, the molecular basis of DIC [87, 88]. In addition, DOX inhibited the expression of genes involved in mitochondrial function and oxidative phosphorylation in the presence of TOPII*β*, such as downregulating the expression of Ndufa3, Sdha, and Atp5a1, which are involved in the electron transport chain, as described above, and induced mitochondrial ultrastructural changes. This may be due to the DOX-TOPII*β* complex binding to the PGC-1*α*/*β* promoter and thereby inhibiting its expression [68]. PGC-1*α* is a major regulator of mitochondrial biogenesis that interacts with nuclear transcription factors to promote the expression of transcription factors required for mtDNA replication, thereby enhancing mitochondrial biogenesis. DOX can downregulate the expression of PGC-1*α* and its downstream signals, such as nuclear respiratory factor 1 (NRF-1), mitochondrial transcription factor A (TFAM), and mitochondrial uncoupling protein 2 (UCP2), by inhibiting AMPK, which has been known to play an essential role in maintaining redox homeostasis, endoplasmic reticulum, and mitochondrial homeostasis in cells, resulting in the reduction and oxidation of mtDNA [89–91]. In addition, DOX can combine with TOPII*β* to induce mtDNA damage, resulting in activation of poly adenosine diphosphate ribose polymerase (PARP) and depletion of intracellular NAD^+^ and ATP. Eventually, glycolysis and mitochondrial respiration rates are slowed [92, 93]. DOX downregulates the expression of the mitochondrial enzyme NAD^+^-dependent deacetylase 3 (SIRT3), thereby increasing mtDNA damage and ROS production and inhibiting mitochondrial respiration [55]. Studies have also shown that ROS production depends on TOPII*β*. DOX treatment increases the production of ROS, which promotes the release of calcium from sarcoplasmic reticulum (SR) and the damage of myocardial cells of calcium removal system to increase levels of calcium in cells. Overloading of mitochondrial calcium causes mitochondrial permeability transition, leading to mitochondrial membrane potential losing, mitochondrial swelling, rupture, and the release of Cytc and apoptosis-inducing factors, which trigger mtDNA damage. Increased calcium, in turn, induces ROS production through calcium-sensitive ROS-producing enzymes, thus forming a vicious cycle [94–96]. Currently, dexrazoxane, the only drug approved by the Food and Drug Administration (FDA) for DIC prevention, prevents double chain rupture by combining with iron chelates to target TOPII*β* or promote degradation of TOPII*β*, thereby improving DIC, suggesting a specific role for this mechanism. However, dexrazoxane still failed to meet the expectations of preclinical studies and its clinical use has been limited by reason of serious adverse reactions such as bone marrow suppression [97, 98]. Therefore, further study and development of drugs targeting TOPII*β* with few toxic side effects is very important. Collectively, it is obvious that the accumulation of mtDNA damage links with the progression of DIC.

### 4.3. Key Receptors, Kinases, and Transcription Factors

Protease-activated receptor 1 (PAR-1), a G-protein-coupled receptor, participates in cardiac injury and adverse remodelling [99]. DOX has been found to activate PAR-1, resulting in increased ROS production, mitochondrial membrane potential losing, and bioenergy impairment in cardiomyocytes and fibroblasts [100]. GATA-4, a key transcription factor in cardiac development, activates the antiapoptosis gene Bcl-XL to regulate apoptotic pathways [94]. Dox inhibits the expression of the mitochondrial GATA-4 gene, thereby inhibiting mitochondrial synthesis and metabolism [72]. Caspase-3 and Caspase-9 are major biomarkers for mitochondrial apoptosis. DOX activates cardiac myocyte p53 through the ERK pathway and upregulates the expression of BAX, thus inducing myocardial mitochondrial apoptosis through Caspase-3 and Caspase-9 [101]. In addition, DOX upregulates the expression of the p53 gene, which binds to the Parkin and inhibits the autophagy clearance of the damaged mitochondria, resulting in mitochondrial biological energy depletion [102]. Lysosomal signalling and function are governed by transcription factor EB (TFEB). Loss of TFEB inhibits lysosomal function and lysosomal autophagy, inducing cardiomyocytes susceptible to DiMBc [103]. In addition, studies have proved that TFEB downregulation is associated with dynamin-related protein 1 (DRP1) and mTOR, and phosphorylation of mTOR is known to inhibit TFEB expression. DRP1 is required for fission of mitochondria and peroxisomes. DOX can inhibit DRP1 phosphorylation and TFEB expression and upregulate mTOR phosphorylation, while MDIVI-1, a selective inhibitor of DRP1, further upregulates mTOR phosphorylation and inhibits TFEB expression. These results suggest that DOX promotes the phosphorylation of mTOR and inhibits the expression of TFEB by inhibiting DRP1 phosphorylation, resulting in the interruption of mitochondrial autophagy, excessive ROS production, and damage to mitochondrial function [104–106]. Previous studies have demonstrated that antioxidant enzymes can protectively detoxify ROS/RNS into less active substances. They are also associated with many redox signalling pathways; for example, glutathione peroxidase 4 (GPX4) can inhibit iron-dependent lipid peroxidation [5, 107]. DOX administration results in significantly reduced glutathione levels and the activity of antioxidant enzymes such as catalase, and superoxide dismutase [108]. Overall, these studies may promise therapeutic targets for preventing DIC.

## 5. Drug Intervention

Currently, there are no specific treatments to prevent or cure DOX-induced cardiotoxicity, and few cardioprotective drugs are trialled in patients for treatment of DIC and these drugs are limited to standard heart failure medications. The only drug approved by FDA which specific for DIC is dexrazoxane. Dexrazoxane is an iron-chelating agent targeting oxidative stress. However, it has failed to achieve the desired effect from preclinical studies while also presenting concerns about its safety [109, 110]. A substantial list of compounds has been shown to alleviate DOX-mediated mitochondrial bioenergetics disorders and is summarized below.

### 5.1. Chemical Drug or Active Substance

Studies have confirmed that some chemical drugs such as hypoglycemic drugs, calcium antagonists, antioxidants, redox modulators, iron chelators, and some related receptor antagonists can prevent DIC [111]. Metformin has a hypoglycemic effect and is widely used to treat type 2 diabetes [112]. Studies have shown that metformin has a protective effect on DOX-mediated mitochondrial damage in mice by activating the AMPK pathway and reducing H_2_O_2_ levels [43, 94]. As a nonselective *β*-blocker, carvedilol has been extensively used in the clinical treatment of hypertension and chronic heart failure. Studies have shown that carvedilol can inhibit DOX-induced oxidative stress and inhibit CI, thereby reducing the production of semiquinone-doxorubicin [113]. Statins rely on RNS and RAS-related C3 botulinum toxin substrate 1 (Rac1) to activate the AMPK pathway in the myocardium [43]. Although RNS adversely affects the myocardium, NO is indispensable for the integrity of cardiovascular function. Supplementation with nitrate, the primary storage form of NO in vivo, has been shown to enhance the activity of CI and its NADH dehydrogenase and counteract the decline in DOX-induced mitochondrial oxidative phosphorylation [114]. It has been reported that LCZ696, a novel angiotensin receptor antagonist, can restore mitochondrial structure and morphology, improve mitochondrial CI activity, and increase ATP production in DOX-induced dilated cardiomyopathy mice by inhibiting dynein-associated protein 1 (Drp1)-mediated mitochondrial dysfunction [105]. EMPA, an SGLT2 inhibitor, has been shown to have a protective effect on DOX-treated mice and H9C2 cardiomyocytes, increasing cell viability, improving mitochondrial dysfunction, and increasing intracellular ATP levels [115]. It has been reported that in cells dexrazoxane, it can be turned into a ring-opening chelating agent, which can replace the DOX-Fe^3+^ complex and bind to iron, interfering with iron-mediated ROS production and blocking the inactivation of respiratory enzymes by the iron complex [64]. Tedesco et al. reported that a novel original formulation named *α*5 consisting of essential amino acids, precursors of the tricarboxylate cycle, and a cofactor promotes mitochondrial biogenesis and anti-ROS production by activating the Akt/eNOS/mTORC1 signalling axis, preventing DOX-induced mitochondrial damage [116]. The development of these chemical agents or active ingredients has greatly improved the therapeutic efficacy of DOX and has provided more possibilities for addressing adverse prognoses from DOX.

### 5.2. Traditional Herbal Medicine or Biologically Active Ingredients

In addition to chemical drugs, many studies have shown that traditional herbal medicine or biologically active ingredients have an attractive protective effect against DIC, and many studies have shown that some herbal medicines can improve the mitochondrial bioenergy disorders caused by DOX (Table 1). Resveratrol can activate the AMPK pathway, reducing DOX-induced ROS levels and improving antioxidant levels [108]. In addition, the natural analogue of resveratrol, taxane, prevents DIC by enhancing AMPK and SIRT1 cascade reactions, activating PGC-1*α*, and thereby reducing oxidative stress [93]. Allicin, the active ingredient of *garlic*, can combat oxidative damage and heart cell apoptosis caused by the inactivation of DOX-mediated antioxidants such as catalase and superoxide dismutase [117]. Cryptotanshinone is one of the primary bioactive constituents isolated from *Salvia miltiorrhiza* and ameliorates DIC by targeting the Akt-GSK-3*β*-mPTP pathway in vitro [81]. Curcumin, a natural compound extracted from *turmeric*, has anti-inflammatory effects. Studies have shown that curcumin upregulates the PI3K/Akt/mTOR pathway, which is essential for cell survival and differentiation and has a regulatory effect on DOX-induced cardiac metabolic remodelling [108]. Luteolin, an active substance extracted from vegetables and fruits, has been shown to improve DOX-induced mitochondrial dysfunction through a Drp1/mTOR/TFEB-dependent mechanism [104]. Ferruginol, isolated from *Salvia*, may promote FAO and improve mitochondrial bioenergy by upregulating the expression of the deacetylases SIRT1 and PGC-1*α* [118]. Harpagoside, a monomer of *Scrophularia ningpoensis*, was reported to improve DiMBc via P53-Parkin-mediated mitophagy [119]. In addition, other studies have shown that Honokiol [69], Schisandrin B [120], Berberine [121], and Compound Danshen Dripping Pill [122] have a protective effect on the heart and can reverse the damage to mitochondrial biological function caused by DOX. A growing number of studies have reported that traditional herbal medicines can regulate DOX-induced myocardial mitochondrial bioenergy disorder and protect the heart (Table 1). Other compounds not classically related to mitochondrial bioenergy have been demonstrated to have cardioprotective effects on DIC. For example, a previous study has shown that tanshinone IIA may restore the dynamic balance of autophagosomes/autolysosomes in DIC by targeting Beclin1/LAMP1 [123]. Dihydrotanshinone I, another natural product from *Salvia miltiorrhiza*, as a novel cardioprotective compound, it could react in the anti-inflammation management of DIC via the mTOR-TFEB-NF-*κ*B signalling pathway [124]. In summary, plentiful evidence indicates the effectiveness of traditional herbal medicine in preventing DIC, a basis for further research into the development of traditional herbal medicine compounds that can intervene in DIC with multiple targets, better effects, and fewer adverse reactions.

## 6. Future Perspectives

Although DOX induces severe cardiotoxicity, including left ventricular dysfunction, cardiomyopathy, arrhythmias, and heart failure [5, 125], it remains the dominant anthracycline in the treatment of a series of cancers due to its high efficacy at low doses, a wide spectrum of antineoplastic effects, and lethality to various tumorous cells with various growth cycle effect advantages [3, 126]. Studies have been carried out to develop more appropriate interventions and treatment strategies for patients receiving anthracycline chemotherapy. A new view suggests that cardiometabolic alterations can be used not only as an early marker for iatrogenic cardiac injury but also as a target for drug intervention [17]. The exact mechanism of DIC is still unclear; here, the mechanism of DiMBc is systematically elucidated, providing an up-to-date source for experimental studies. Furthermore, the roles of oxidative stress and autophagy in DIC have been confirmed but the pathways of intracellular redox reactions and cell death are complex and interchangeable and the exact relationship between them and energy metabolism remains to be further explored. Regarding the treatment of DIC, many studies have described DOX-mediated cardiometabolic changes in pharmacological therapy, including imidazolidine, natural extracts, animal extracts, and synthetic artificial antioxidants [82], but the effects of many active ingredients remain to be clinically validated. In addition, advances have been made in bioenergy-based preventive therapies. As a natural library for drug molecular screening, traditional herbal medicine compounds can potentially aid the prevention and treatment of DIC; thus, the development of drugs targeting biological energy based on traditional herbal medicine has broad prospects. However, few solid preclinical and clinical studies have been performed to date and it remains necessary to conduct in-depth research and develop drugs to prevent and treat DIC more effectively.

## Figures and Tables

**Figure 1:** Multiple mechanisms of doxorubicin-induced myocardial mitochondrial bioenergetics disorder.

**Figure 2:** Doxorubicin-induced myocardial mitochondrial substrate metabolism disorder. Abbreviations. AKT: serine/threonine kinase; GLUT1: glucose transporter 1, IFN*γ*: interferon gamma; IFN*γ*R: interferon gamma receptor; AMPK: adenosine 5′-monophosphate (AMP)-activated protein kinase; ACC: acetyl-CoA carboxylase; ERK: extracellular regulated protein kinases; FAO: fatty acid oxidation; CPT1: carnitine palmitoyltransferase 1; PFK phosphofructokinase; CS citrate synthase.

**Figure 3:** Doxorubicin disturbs the myocardial mitochondrial respiratory chain and the storage/utilization of ATP. Abbreviations. SQ-DOX: doxorubicin semiquinone type; ROS: reactive oxygen species; RNS: reactive nitrogen species; Cytc: cytochrome c; COX1: complex IV subunit 1; UCP3: mitochondrial uncoupling protein 3; Bnip3: Bcl-2/19-kDa interaction protein 3; Ndufa: NADH ubiquinone oxidoreductase subunit A3; Sdha: succinate dehydrogenase complex flavoprotein subunit A; Atp5a1: ATP synthase, H^+^ transporting, mitochondrial F1 complex, alpha subunit 1; ΔΨm: mitochondrial membrane potential.

**Figure 4:** Other mechanisms by which DOX affects myocardial mitochondrial bioenergy. Abbreviations. VDAC: voltage-dependent anion channels; ANT: adenine nucleotide (ADP/ATP) translocator; NF-*κ*B: nuclear factor kappa-B; Bnip3: Bcl-2/19-kDa interaction protein 3; AIF: apoptosis inducing factor; DRP1: dynamin-related protein 1; NRF-1: nuclear respiratory factor 1; TFAM: mitochondrial transcription factor A; UCP2: mitochondrial uncoupling protein 2; GATA-4: GATA-binding protein 4; PGC-1*α*: peroxisome proliferator-activated receptor-gamma coactivator (PGC)-1alpha.

**Table 1:** Herbal medicine and its small molecules that target mitochondria effectively prevent DIC.

Molecules	Study model	Methods (drug/dose/route/duration)	Key mechanisms against dox-induced mitochondrial biogenetics disorder	Refs

Chrysin	SD rats	(i) Chr/50 mg/kg/4 times/w/ig/4 w+dox/5 Mg/kg/w/ip/4 w	Oxidative stress↓	[127]
			p53↓	
			Mito-apoptotic pathway↓	

Tetrandrine	C57 mice	(i) Tet/50 mg/kg/d/po/4 d+dox/15 mg/kg/single dose/ip/3 d (start 1 d after Tet)	Nrf-2↑	[128]
			Oxidative stress↓	

*Irvingia gabonensis*	Wistar rats	(i) IGESE/100 mg/kg/d/po/13 d+dox/15 mg/kg/single dose/ip/3 d (start 10 d after IGESE)	Oxidative stress↓	[129]
			Serum lipids↓	

*Hippophae rhamnoides* (alk-A, alk-B)	H9C2 cells	(i) Alk-A, alk-B/10,20,40 *μ*M/25 h+dox/2.5 *μ*M/24 h (start 1 h after alk)	Oxidative stress↓	[130]
			caspase3↓	
			mtDNA damage↓	
			ATP↑	

Compound Danshen Dripping Pill	C57 mice	(i) CDDP/660,2640 mg/kg/d/po/31 d+dox/2 mg/kg/7 d/ip/28 d (start 3 d after CDDP)	Nrf-2↑	[122]
			p-AMPK↑	
			HK↑	
			CS↑	

Licorice root extract	H9C2 cells	(i) Gg/40 *μ*g/ml/24 h+dox/5 *μ*M/24 h	Oxidative stress↓	[131]
			Disruption of ΔΨm↓	
			Lipid accumulation↓	
			SIRT-1/PPAR*γ*↑	

Shenmai injection	H9C2 cells	(i) SMI/0.5%,0.25%/24 h+dox/1 *μ*M/16 h (start 8 h after SMI)	Mito-superoxide anion↓	[132]
			Disruption of ΔΨm↓	
			Mitochondrial fragmentation↓	
			p-AMPK↑	
			p-DRP1↑	
			Mito-respiratory dysfunction↓	

Cryptotanshinone	H9C2 cells	(i) Cts/5,10,25 *μ*M/48 h+dox/1 *μ*M/24 h (start 24 h after Cts)	Oxidative stress↓	[81]
			Mito-apoptotic pathway↓	
			Disruption of ΔΨm↓	
			p-GSK-3*β*-ANT interaction↑	
			ANT-CypD complex↓	

Astragali Radix	H9C2 cells	(i) AR/400-1600 *μ*g/ml/30 h+dox/0.5 *μ*M/24 h (start 6 h after AR)	Fatty acid metabolism↑	[133]
			PPAR*γ*↑	

Esculetin	H9C2 cells	(i) Dox/8 *μ*M/24 h+Esc/10 *μ*M/2 h	caspase3↓	[134]
			PARP↓	
			Oxidative stress↓	

Curcumin	Wistar rats H9C2 cells	(i) Dox/40 mg/kg/single dose/ip + Cur/100 mg/kg/d/po/7 d(start 5 d after dox) (ii) Cur/20 *μ*M/48 h+dox/15 *μ*M/24 h (start 24 h after Cur)	Oxidative stress↓	[135, 136]
			caspase3↓	
			Uphold mitochondrial integrity	

Honokiol	C57 mice NRCMs	(i) HKL/0.2 mg/kg/d/ip/5 w+dox/5 mg/kg/w/ip/4 w (start 1 week after HKL) (ii) dox/2 *μ*M/24 h+HKL/10 *μ*M/24 h	Mito-respiratory dysfunction↓	[33, 55]
			Oxidative stress↓	
			PPAR*γ*↑	
			Oxidative stress↓	
			mtDNA damage↓	
			Citrate synthase activity↑	
			SIRT-3↑	

Matrine	C57 mice H9C2 cells	(i) Dox/4 mg/kg/w/ip/4 w+Mat/200 mg/kg/d/ig/4 w (ii) Mat/200 *μ*M/L/24 h+dox/1 *μ*M/L/24/h	Oxidative stress↓	[137]
			Mito-apoptotic pathway↓	
			AMPK*α*/UCP2↑	

Berberine	SD rats H9C2 cells	(i) Ber/10,20 mg/kg/d/po/16 d+dox/20 mg/kg/2 d/ip/6 d (start 11 d after Ber) (ii) Ber/0.1,1,10 *μ*M/48 h + dox/1 *μ*M/24 h (start 24 h after Ber)	Oxidative stress↓	[121]
			Disruption of ΔΨm↓	
			Mitochondrial Ca^2+^ overload↓	
			SIRT-1↑	

Salidroside	C57 mice NRCMs	(i) SAL/180 mg/kg/d/ig/8 w+dox/5 mg/kg/w/ip/5 w (start 3 weeks after SAL) (ii) SAL/100 *μ*M/L/48 h+dox/1 *μ*M/24 h (start 24 h after SAL)	Oxidative stress↓	[138]
			caspase3↓	

Liensinine	Mice NMVMs	(i) LIEN/60 mg/kg/single dose/ip/6 d+dox/5 mg/kg/single dose/ip/6 d (ii) LIEN/20 *μ*M/24 h+dox/5 *μ*M/24 h	Mito-aconitase activity↑	[139]
			Mito-respiratory dysfunction↓	
			Disruption of ΔΨm↓	
			Oxidative stress↓	
			Mitochondrial fission↓	
			ERK/DRP1↓	
			Mitophagy↓	

Yellow wine polyphenolic compounds	SD rats H9C2 cells	(i) YWPC/30 mg/kg/d/ig/4 w+dox/3 mg/kg/3 times/w/2 w (ii) YWPC/50 mg/L/24 h+dox/5 *μ*M/L/24 h	Oxidative stress↓	[140]
			Uphold mitochondrial integrity	
			Disruption of ΔΨm↓	
			caspase3↓	
			Nucleus Nrf-2↑	

Epigallocatechin-3-gallate	C57 mice NRCMs H9C2 cells	(i) Dox/2.5 mg/kg/2 times/w/ip/3 w+EGCG/20 mg/kg/d/ig/6 w (start 1 h after dox) (ii) EGCG/20 *μ*M/72 h+dox/1 *μ*M/48 h (start 24 h after EGCG)	AMPK*α*2↑	[141]
			TCA cycle↑	
			Oxidative stress↓	
			Lipid metabolism↑	
			Mito-respiratory dysfunction↓	
			Disruption of ΔΨm↓	
			Mitochondrial iron overload↓	

Cardamonin	C57 mice HL-1 cells	(i) CAR/20,40,80 mg/kg/d/ig/4 w+dox/5 mg/kg/w/ip/4 w (ii) CAR/50,100 *μ*M/24 h+dox/5 *μ*M/24 h	Oxidative stress↓	[142]
			Mito-apoptotic pathway↓	

Ferruginol	C57 mice H9C2 cells	(i) Dox/5 mg/kg/1 time/w/iv/4 w+FGL/20 mg/kg/d/ig/4 w (start 1 w after last dose of dox) (ii) FGL/0.1-50 *μ*M/24 h+dox/1 *μ*M/24 h	Mitochondrial biogenesis↑	[118]
			FAO↑	
			Oxidative stress↓	
			SIRT-1/PGC-1*α*↑	
			Disruption of ΔΨm↓	

Harpagoside	Zebrafish C57 mice H9C2 cells	(i) HAR/25 *μ*M/3 d+dox/100 *μ*M/L/3 d (ii) dox/5 mg/kg/1 time/w/iv/4 w+HAR/42 mg/kg/d/po/4 w (start 1 w after last dose of dox) (iii) HAR/1-500 *μ*M/48 h+dox/1 *μ*M/24 h (start 24 h after HAR)	mtDNA damage↓	[119]
			Oxidative stress↓	
			p53↓	
			Parkin↑	
			Mitophagy↑	

↑: increase or activate; ↓: decrease or inhibit; NRCMs: neonatal rat cardiomyocytes; NMVMs: neonatal mouse ventricular myocytes; w: week/weeks; mito-: mitochondrial; ΔΨm: mitochondrial membrane potential; TCA cycle: tricarboxylic acid cycle.

## Data Availability

All datasets (editable figures in PowerPoint format) used to support this study will be made available upon request.
